This article has been retracted.

# MicroRNA-1468 promotes tumor progression by activating PPAR-γ-mediated AKT signaling in human hepatocellular carcinoma

**DOI:** 10.1186/s13046-018-0717-3

**Published:** 2018-03-06

**Authors:** Zhikui Liu, Yufeng Wang, Changwei Dou, Liankang Sun, Qing Li, Liang Wang, Qiuran Xu, Wei Yang, Qingguang Liu, Kangsheng Tu

**Affiliations:** 1 Department of Hepatobiliary Surgery, the First Affiliated Hospital of Xi’an Jiaotong University, 277 Yanta West Road, Xi’an, 710061 China; 2 Department of Hepatobiliary Surgery, Zhejiang Provincial People’s Hospital (People’s Hospital of Hangzhou Medical College), Hangzhou, Zhejiang 310014 China; 3 Key Laboratory of Tumor Molecular Diagnosis and Individualized Medicine of Zhejiang Province, Zhejiang Provincial People’s Hospital (People’s Hospital of Hangzhou Medical College), Hangzhou, Zhejiang 310014 China

**Keywords:** miR-1468, Hepatocellular carcinoma, CITED2, UPF2, PPAR-γ, Tumor growth

## Abstract

**Background:**

Accumulating evidence confirm that aberrant microRNAs (miRNAs) expression contributes to hepatocellular carcinoma (HCC) development and progression. Previous study reported that miR-1468 showed an up-regulated tendency and might be a potential prognostic biomarker in HCC samples derived from TCGA database. However, the role of miR-1468 and its underlying mechanisms involved in the growth and metastasis of HCC remain poorly investigated.

**Methods:**

CCK-8, EdU, colony formation and flow cytometry were used to determine proliferation, cell cycle progression and apoptosis of HCC cells in vitro. The subcutaneous tumor model in nude mice was established to detect tumor growth of HCC in vivo. The direct binding of miR-1468 to 3’UTR of Cbp/p300 interacting transactivator with Glu/Asp rich carboxy-terminal domain 2 (CITED2) and Up-frameshift protein 1 (UPF1) was confirmed by luciferase reporter assay.

**Results:**

Here, we demonstrated that miR-1468 expression was up-regulated in HCC tissues and cell lines. Clinical analysis revealed that increased miR-1468 level was significantly correlated with malignant prognostic features and shorter survival. Gain- and loss-of-function experiments indicated that miR-1468 promoted cell proliferation, colony formation, cell cycle progression and induced apoptosis of HCC cells in vitro and in vivo. Moreover, CITED2 and UPF1 were identified as direct downstream targets of miR-1468 in HCC cells, and mediated the functional effects of miR-1468 in HCC, resulting in peroxisome proliferator-activated receptor-γ (PPAR-γ)/AKT signaling activation. In clinical samples of HCC, miR-1468 inversely correlated with the levels of CITED2 and UPF1, which were confirmed to be down-regulated in HCC. Restoration of CITED2 or UPF1 expression at least partially abolished the biological effects of miR-1468 on HCC cells. Moreover, alteration of PPAR-γ or AKT phosphorylation could reverse the function of miR-1468 in HCC.

**Conclusions:**

Taken together, this research supports the first evidence that miR-1468 plays an oncogenic role in HCC via activating PPAR-γ/AKT pathway by targeting CITED2 and UPF1, and represents a promising therapeutic strategy for HCC patients.

**Electronic supplementary material:**

The online version of this article (10.1186/s13046-018-0717-3) contains supplementary material, which is available to authorized users.

## Background

Hepatocellular carcinoma (HCC) is the fifth most common malignancies worldwide and the second leading cause of cancer-related death which contribute to increasing morbidity and mortality in China according to world health organization (WHO) [1, 2]. Despite great advancement in diagnosis and therapeutic strategy, including novel chemotherapeutic interventions and liver transplantation, the long-term survival remains dismal because of high rate of intrahepatic and distal metastasis [3, 4]. Therefore, it is urgent to elucidate the molecular mechanisms underlying HCC progression and develop promising biomarkers for cancer treatment.

MicroRNAs (miRNAs), a family of small, single-stranded and non-coding evolutionarily conserved RNAs of approximately 21–25 nucleotides in sequence length, act as post-transcriptional modulator of gene expression in cancer progression by interacting with complementary sequences within the 3′-untranslated region (UTR) of target mRNA to induce mRNA degradation or translational repression [5–7]. Increasing evidence confirm that dysregulated miRNAs are involved in various biological processes in HCC [8], including cell proliferation, cell cycle, apoptosis and metastasis [9, 10]. Therefore, miRNAs have been recognized as promising therapeutic and prognostic biomarkers in HCC diagnosis and treatment. MiR-1468, a novel cancer related microRNA, was dysregulated and could predict patients’ survival in diverse cancers [11]. Jiang et al. confirmed that miR-1468 inhibited cell proliferation and induced cell cycle arrest by targeting ribonucleotide reductase large subunit M1 (RRM1) in glioma [12]. In papillary renal cell carcinoma (pRCC), miR-1468 was significantly associated with patient survival and identified by multivariate Cox regression analyses as potential independent prognostic factors in pRCC [13]. In lung adenocarcinoma, miR-1468 expression was significantly correlated with recurrence-free survival [14]. Moreover, miR-1468 was decreased in blood-based microRNA biomarker in early diagnosis of pancreatic cancer [15]. Previous study reported that miR-1468 showed an up-regulated tendency and might be a potential prognostic biomarker in HCC samples derived from The Cancer Genome Atlas (TCGA) database [16]. Nevertheless, the function of miR-1468 and its underlying molecular mechanisms in HCC remain unknown.

Peroxisome proliferator-activated receptor-γ (PPAR-γ) is a ligand-activated transcription factor, which belongs to the nuclear receptor superfamily and exerts its function on tumor promotion, cellular differentiation, cell cycle and apoptosis [17, 18]. In HCC, PPAR-γ has been identified as a tumor suppressor gene and mediated apoptosis of HCC cells depends on modulation of phosphatidylinositol 3-kinase (PI3K) pathway [19, 20]. Moreover, recent findings using PPAR-γ knockout mice suggest that PPAR-γ reduces HCC carcinogenesis and metastasis and acts as a tumor-suppressor gene in the liver [21]. PPAR-γ agonist induces apoptosis by triggering the intrinsic apoptosis pathway and inhibiting PI3K/AKT survival pathway in human cervical cancer cells [22]. Our previous study confirms that miR-130b promotes cell aggressiveness by inhibiting PPAR-γ in human HCC [23]. These findings indicate that PPAR-γ regulates HCC tumorigenesis and progression.

In present research, we demonstrated that miR-1468 overexpression was associated with poor prognostic features and reduced survival of HCC patients. MiR-1468 promoted the growth of HCC cells in vitro and in vivo*.* Furthermore, we confirmed that miR-1468 inhibited PPAR-γ/AKT signaling activity through directly suppression of Cbp/p300 interacting transactivator with Glu/Asp rich carboxy-terminal domain 2 (CITED2) and Up-frameshift protein 1 (UPF1). Therefore, our results confirm that miR-1468 exerts a critical role in HCC progression and represents a potential target for HCC diagnosis and treatment.

## Methods

### Patients’ tissues and cell culture

Patients’ tissues and paired adjacent non-tumor tissues were obtained from 99 patients in our hospital after the informed consent were obtained from all patients. All patients didn’t receive any therapy including radiotherapy, chemotherapy or radiofrequency ablation before surgery. The clinicopathological and demographic information of the patients was described in Table 1. The normal immortalized human hepatocyte LO2 and a panel of HCC cells (Hep3B, HepG2, Huh7, MHCC-97 L and SMMC-7721) (Chinese Academy of Sciences, Shanghai, China) were maintained in DMEM (Invitrogen, Carlsbad, USA) containing 10% FBS (Gibco, GrandIsland, USA) in 37 °C with 5% CO2.

**Table 1:** Clinical correlation of miR-1468 expression in hepatocellular carcinoma (*n* = 99)

Clinical parameters	Number	Expression level		*P* value
		miR-1468^high^(*n* = 50)	miR-1468^low^(*n* = 49)	
Age (years)				
< 50	32	18	14	0.429
≥ 50	67	32	35	
Gender				
Male	73	36	37	0.692
Female	26	14	12	
Tumor size (cm)				
< 5	75	32	43	0.006^*^
≥ 5	24	18	6	
Tumor number				
Solitary	85	53	42	0.684
Multiple	14	7	7	
Edmondson-Steiner grading				
I + II	77	34	43	0.018^*^
III + IV	22	16	6	
TNM stage				
I + II	79	35	44	0.014^*^
III + IV	20	15	5	
Venous infiltration				
Present	15	8	7	0.812
Absent	84	42	42	
AFP (ng/ml)				
< 400	27	15	12	0.538
≥ 400	72	35	37	
HBsAg				
Positive	90	44	46	0.487
Negative	9	6	3	

*AFP* alpha-fetoprotein, *TNM* tumor-node-metastasis

^*^Statistically significant

### Quantitative real-time polymerase chain reaction (qRT-PCR)

qRT-PCR was conducted as reported previously [10, 24, 25]. All RNA was extracted based on the protocol of TRIzol reagent (Invitrogen, Carlsbad, CA, USA). qPCR primer against miR-1468 (HmiRQP0193), U6 (HmiRQP9001), CITED2 (HQP062677), UPF1 (HQP071077) and GAPDH (HQP006940) were ordered from Genecopoeia (Guangzhou, China).

### Immunohistochemical staining (IHC)

The sections were dewaxed, dehydrated, and rehydrated. CITED2, UPF1 (1:100, Cell Signaling, Danvers, MA, USA) were added to the sections and incubating at 4 °C overnight. Then applying the biotinylated secondary antibodies (Goldenbridge, Zhongshan, China) according to SP-IHC assays. Specific experiment was conducted similar to previously reported [24, 26].

### Immunofluorescence (IF)

We used 4% paraformaldehyde to fix transfected cells and used 0.3% Triton X-100 to permeabilize. The primary antibody CITED2 (Novous Biologicals, Inc. Littleton, CO, USA), UPF1 (Cell Signaling Technology, Danvers, USA) was used. Then the Alexa Fluor-conjugated secondary antibody was performed the next experiment. Lastly, the images were taken by Microscope (Zeiss, Germany).

### Western blot analysis

We separated proteins by SDS–PAGE and transferred proteins to PVDF membranes. Detailed experiment was performed similar to previously reported [24, 26].

### RNA interference transfection

The CITED2, UPF1 and a negative control siRNA were synthesized by GenePharm (Shanghai, China). Hep3B and MHCC-97 L cells (2 × 10^5^ per well) were transfected in a concentration of 100 nM siRNA.

### Cell proliferation, cell cycle and apoptosis detection

Cell Counting Kit-8 (CCK8) reagents (Dojindo, Kumamoto, Japan), EdU, cell cycle, colony formation and apoptosis were carried as described previously [10, 27].

### Luciferase reporter assay

The 3’-UTR sequence of CITED2 and UPF1, together with a corresponding mutated sequence within the predicted target sites, were synthesized and inserted into the pmiR-GLO dual-luciferase miRNA target expression vector (Promega, Madison, WI, USA). The assays were carried out as described previously [10, 28].

### In vivo experiments

Four-to-six-week-old male BALB/c nude mice (Centre of Laboratory Animals, The Medical College of Xi’an Jiaotong University, Xi’an, China) were used to establish the nude mouse xenograft model. Hep3B (5 × 10^6^) cells that were transfected with miR-1468 or miR-control vectors or MHCC-97 L cells with anti-miR-1468 were mixed in 150 μl of Matrigel and were inoculated subcutaneously into the flank of nude mice. The tumor volume for each mouse was determined by measuring two of its dimensions and then calculated as tumor volume = length × width × width/2. After 3 weeks, the mice were sacrificed by cervical dislocation under anesthesia with ether and the xenograft tumor tissue was explanted for examination. Animal protocols were approved by the Institutional Animal Care and Use Committee of Xi’an Jiaotong University.

### Statistical analysis

Results are managed as the mean ± SD and analyzed by SPSS software, 16.0 (SPSS, Chicago, USA). The statistical approaches mainly included a two-tailed Student’s t test, a Kaplan–Meier plot, Pearson chi-squared testand so on. Difference with *P* < 0.05 was regard to be significant. Graphs were mainly made by GraphPad Prism 6 (GraphPad, San Diego, USA).

## Results

### miR-1468 is up-regulated in HCC and correlates with patients’ survival

To explore the expression level of miR-1468 in HCC, we performed qRT-PCR to measure its expression in 40 pairs of randomly selected tumor tissues and matched adjacent non-tumor tissues. We found that miR-1468 was significantly up-regulated in HCC tissues compared with matched non-tumor tissues (*P* < 0.05, Fig. 1a). Similarly, miR-1468 was obviously increased in a group of HCC cell lines as compared with normal hepatic cell line LO2 (*P* < 0.05, respectively, Fig. 1b). Next, we divided all HCC patients into miR-1468 high (*n* = 50) and low (*n* = 49) group according to median value. As shown in Table 1, increased miR-1468 level was markedly associated with large tumor size (≥5 cm; *P* = 0.006), high histological grade (Edmondson-Steiner grade III + IV; *P* = 0.018) and advanced tumor stage (TNM stage III + IV; *P* = 0.014). Furthermore, Kaplan-Meier analysis revealed that HCC patients with high miR-1468 level showed a significant shorter overall survival (*P* = 0.0004, Fig. 1c) and disease-free survival (*P* = 0.0006, Fig. 1d). In addition, miR-1468 was an independent factor for predicting 5-year overall and disease-free survival in HCC patients (*P* = 0.003 and 0.007, respectively, Table 2). Our data indicates that miR-1468 may server as a novel predictive biomarker for HCC patients.

**Fig. 1:** MiR-1468 is down-regulated in HCC and correlates with HCC progression and survival. Comparing differences in the expression of miR-1468 between (**a**) HCC and matched tumor-adjacent tissues and (**b**) HCC cell lines and the immortalized hepatic cell line LO2. HCC patients with higher expression of miR-1468 had worse overall survival (**c**) and disease-free survival (**d**). *P < 0.05, **P < 0.01

**Table 2:** Multivariate Cox regression analysis of 5-year overall and disease-free survival of hepatocellular carcinoma patients

Variables	Overall survival			Disease-free survival		
	HR	95% CI	*P*	HR	95% CI	*P*
miR-1468	4.762	1.756–11.482	0.003^*^	3.854	1.527–9.485	0.007^*^
Tumor size	2.745	1.249–5.898	0.012^*^	2.212	1.153–4.675	0.014^*^
Edmondson-Steiner grading	2.168	1.102–4.254	0.018^*^	3.612	1.119–4.856	0.008^*^
TNM stage	3.328	2.245–5.989	0.001^*^	3.478	2.241–6.345	0.010^*^

*TNM* tumor-node-metastasis, *HR* hazard ratio, *CI* confidence interval

^*^statistically significant

### miR-1468 promotes cell growth and inhibits apoptosis of HCC cells

To further investigate the biological function of miR-1468 in HCC, miR-1468 was stably overexpressed in Hep3B cells by lentivirus system and knocked down in MHCC-97 L cells, which contained different endogenous miR-1468 levels. As measured by qRT-PCR, we confirmed that miR-1468 was effectively upregulated in Hep3B or downregulated in MHCC-97 L cells (*P* < 0.05, Fig. 2a). CCK8 and EdU proliferation assays found that miR-1468 overexpression enhanced cell proliferation (*P* < 0.05, Fig. 2b, c). The colony formation assay revealed that ectopic expression of miR-1468 significantly increased cell colonies (*P* < 0.05, Fig. 2d). As determined by flow cytometry, overexpression of miR-1468 promoted cell cycle transition from G1 to S phase (*P* < 0.05, Fig. 2e) and apoptosis resistance (*P* < 0.05, Fig. 2f). In addition, immunoblotting analysis confirmed that up-regulated miR-1468 level obviously increased Cyclin D1 and Bcl-2 expression, while reduced the levels of p21 and Bax (*P* < 0.05, respectively, Fig. 2g). In accordance, miR-1468 knockdown inhibited the growth and induced apoptosis of MHCC-97 L cells (*P* < 0.05, Fig. 2b-g). Thus, these data demonstrate that miR-1468 regulates HCC cell proliferation, cell cycle progression, colony formation and apoptosis in vitro.

**Fig. 2:** MiR-1468 promotes cell proliferation, cell cycle progression, colony formation and inhibits apoptosis in HCC cells in vitro. **a** Hep3B and MHCC-97 L cells that were transfected with corresponding miRNA vectors were subjected to qRT-PCR for miR-1468 expression. Overexpression of miR-1468 promoted cell proliferation (**b**, **c**), colony formation (**d**), cell cycle progression (**e**) and inhibited apoptosis (**f**) in Hep3B cells, while down-regulation of miR-1468 inhibited cell proliferation (**b**, **c**), colony formation (**d**), cell cycle progression (**e**) and promoted apoptosis (**f**) in MHCC-97 L cells. **g** Western blot analysis of cycle regulator Cyclin D1 and p21, apoptosis-related protein Bcl2/Bax expression in the presence and absence of miR-1468. n = six independent experiments. *P < 0.05, **P < 0.01

To measure the effect of miR-1468 on cell tumorigenicity in vivo, we established a subcutaneous tumor model. The tumor growth curves revealed that miR-1468 overexpression significantly promoted the tumor growth, while miR-1468 knockdown inhibited the tumor growth of HCC cells in mice (*P* < 0.05, Fig. 3a). Next, we evaluated the proliferative and apoptotic rate in vivo by Ki67 and TUNEL staining in the xenografted tissues. As expected, miR-1468 overexpression increased the number of Ki67 positive staining cells and reduced the number of apoptotic cells (*P* < 0.05, Fig. 3b, c). However, miR-1468 knockdown inhibited proliferation and induced apoptosis in vivo (*P* < 0.05, Fig. 3b, c). Taken together, these results demonstrate that miR-1468 promotes tumor growth of HCC in vitro and in vivo.

**Fig. 3:** MiR-1468 promotes tumor growth and inhibits apoptosis in vivo. **a** Representative pictures of HCC xenografts from both Hep3B-miR-1468 (left panel) and MHCC-97 L-anti-miR-1468 cells (right panel). Tumor growth curve revealed that miR-1468 overexpression significantly promoted, while miR-1468 knockdown inhibited tumor growth in vivo. Tumor nodules were subjected to immunohistochemical staining for Ki-67 (**b**) and TUNEL (**c**) assays and quantitative analysis. Representative immunostaining and TUNEL assays revealed that miR-1468 overexpression significantly increased the number of Ki-67 positive cells and inhibited the number of apoptotic cells. However, the percentage of Ki-67 positive cells in tumors arising from the miR-1468 knockdown group was significantly lower and the percentage of apoptotic cells was significantly higher than that in the negative control (NC) group. *P < 0.05

### CITED2 and UPF1 are downstream targets of miR-1468 in HCC

We used target algorithm (TargetScan and miRNAda) to predict candidate targets of miR-1468 and found that the 3’-UTR of CITED2 and UPF1 matched the “seed sequence” of miR-1468 (Fig. 4a). Luciferase reporter assay showed that miR-1468 overexpression inhibited, while miR-1469 knockdown increased the luciferase activity of wild-type (wt) CITED2 or UPF1 3’-UTR but not the mutant (mt) CITED2 or UPF1 3’-UTR (*P* < 0.05, Fig. 4b). Furthermore, miR-1468 overexpression significantly inhibited the mRNA and protein expression of CITED2 and UPF1 in Hep3B cells (*P* < 0.05, respectively, Fig. 4c, d). By contrast, the expression of CITED2 and UPF1 were significantly increased by miR-1468 knockdown in MHCC-97 L cells (*P* < 0.05, respectively, Fig. 4c, d). In addition, IF data further confirmed the above results (Fig. 4e, f). These results reveal that miR-1468 inhibits CITED2 and UPF1 expression by directly binding to their 3’-UTR.

**Fig. 4:** CITED2 and UPF1 are direct targets of miR-1468 in HCC cells. **a** miR-1468 and its putative binding sequences in the 3’-UTR of CITED2 and UPF1. The mutant binding site was generated in the complementary site for the seed region of miR-1468. **b** miR-1468 overexpression significantly suppressed, while miR-1468 loss increased the luciferase activity that carried wild-type (wt) but not mutant (mt) 3’-UTR of CITED2 or UPF1. **c** Hep3B and MHCC-97 L cells that were transfected with precursor miR-1468 and miR-1468 inhibitors (anti-miR-1468), respectively, were subjected to qRT-PCR for CITED2 and UPF1 mRNA expression. **d** miR-1468 overexpression reduced the expression of CITED2 and UPF1 protein in Hep3B cells and miR-1468 knockdown increased the level of CITED2 and UPF1 protein in MHCC-97 L cells. **e**, **f** Immunofluorescence staining of CITED2 and UPF1 after transduction of miR-1468. n.s, no significance, *P < 0.05

### miR-1468 inversely correlates with CITED2 and UPF1 expression in HCC tissues

Next, we measured the expression of CITED2 and UPF1 in different miR-1468 groups. Our data revealed that both CITED2 and UPF1 levels in HCC tissues with high miR-1468 level were significantly lower than those in low miR-1468 group (*P* < 0.05, Fig. 5a, b). Moreover, we found that the mRNA level of CITED2 and UPF1 was inversely correlated with miR-1468 expression in the HCC tissues (R^2^ = 0.5753 and 0.5636, *P* < 0.0001, Fig. 5c). Consistently, CITED2 and UPF1 protein expression in miR-1468 high-expressing tumors were obviously lower than those in miR-1468 low-expressing tumors as suggested by IHC, and both CITED2 and UPF2 staining were weaker than adjacent nontumor tissues (*P* < 0.05, Fig. 5d). In addition, western blot demonstrated that CITED2 and UPF1 were significantly down-regulated in HCC tissues compared with matched non-tumor tissues (*P* < 0.05, Fig. 5e). We further evaluated the expression of CITED2 and UPF1 in xenografted tissues and found that miR-1468 overexpression group showed a weak CITED2 and UPF1 staining, however, miR-1468 knockdown group showed opposite effects (*P* < 0.05, Fig. 5f). Taken together, these data suggest that CITED2 and UPF1 expression are inversely associated with miR-1468 in HCC tissues.

**Fig. 5:** An inverse correlation between miR-1468 and CITED2, UPF1 expression is observed in HCC tissues. **a** and **b** The expression of CITED2 and UPF1 in miR-1468 high-expressing tumors was significantly lower than that in miR-1468 low-expressing tumors, as determined by qRT-PCR and immunoblotting. **c** An inverse correlation between the levels of miR-1468 and CITED2, UPF1 mRNA was observed in HCC tissues. **d** Representative immunohistochemical staining showed a weak staining of CITED2, UPF1 in miR-1468 high-expressing HCC tissue and strong staining of CITED2, UPF1 in the miR-1468 low-expressing tumor. The adjacent nontumor tissues show a stronger staining of CITED2 and UPF1 compared to HCC tissues. **e** The expression of CITED2 and UPF1 were down-regulated in HCC tissues compared with matched non-tumor tissues. **f** Xenografts tissues immunohistochemical staining of CITED2 and UPF1 in miR-1468 overexpression or knockdown subcutaneous tumor nodules. *P < 0.05

### Restoration of CITED2 and UPF1 reverses the biological effects of miR-1468 on HCC cells

To investigate the importance of CITED2 and UPF1 in the biological function of miR-1468 in HCC cells, CITED2 or UPF1 was respectively restored in miR-1468-overexpressing Hep3B cells, and inhibited by corresponding siRNA in miR-1468-suppressive MHCC-97 L cells (*P* < 0.05, Fig. 6a). CITED2 or UPF1 restoration reversed the promotive effects of miR-1468 on cell proliferation (P < 0.05, Fig. 6b, c), colony formation (*P* < 0.05, Fig. 6d), cell cycle progression (*P* < 0.05, Fig. 6e) and apoptosis (P < 0.05, Fig. 6f). Moreover, CITED2 or UPF1 knockdown abolished the inhibitory effects of miR-1468 inhibition on HCC cells (*P* < 0.05, Fig. 6b-f). In addition, alteration of CITED2 or UPF1 expression also abolished the effects of miR-1468 on cell cycle and apoptosis-related protein (*P* < 0.05, Fig. 6g). Moreover, inhibition of CITED2 or UPF1 mimics miR-1468-induced effects in control cells (Additional file 1: Figure S1). These results confirm that CITED2 and UPF1 are functional mediators of miR-1468 in HCC cells.

**Fig. 6:** Modulation of CITED2 or UPF1 partially abolishes miR-1468-mediated cellular processes in HCC. **a** miR-1468-overexpressing Hep3B cells that were transfected with empty vector (EV) or CITED2, UPF1 overexpression plasmid were subjected to western blot for CITED2 and UPF1. miR-1468-suppressive MHCC-97 L cells that were transfected with scrambled siRNA or CITED2, UPF1 siRNA were subjected to western blot for CITED2, UPF1. CITED2 or UPF1 restoration abrogated the effects of miR-1468 overexpression on cell proliferation (**b**, **c**), colony formation (**d**), cell cycle progression (**e**) and apoptosis (**f**) of Hep3B cells. CITED2 or UPF1 knockdown reversed the suppressive effects of miR-1468 knockdown in MHCC-97 L cells (**b**-**f**). **g** Alteration of CITED2 or UPF1 abolished the effects of miR-1468 on cell cycle and apoptosis associated factors. *P < 0.05

### PPAR-γ/AKT signaling is essential for the biological function of miR-1468 in HCC

Previous studies confirm that the target genes of miR-1468 are significantly enriched in PPAR signaling pathway and CITED2 is involved in PPAR-γ effects on HCC growth [16, 29]. Therefore, we explored the PPAR-γ/AKT signaling by western blot. As shown in Fig. 7a, overexpression of miR-1468 significantly inhibited, while miR-1468 knockdown promoted PPAR-γ/AKT pathway in HCC cells (*P* < 0.05, Fig. 7a), with change of p-AKT level rather than total AKT (*P* < 0.05, Fig. 7a). Moreover, CITED2 or UPF1 overexpression promoted PPAR-γ/AKT pathway in HCC cells (Additional file 2: Figure S2). To investigate whether PPAR-γ mediated miR-1468-induced biological function in HCC cells, we treated miR-1468-overexpressing Hep3B cells with the agonist rosiglitazone (40 μM). We found that rosiglitazone at least partially inhibited miR-1468-induced cell proliferation, cell cycle progression, colony formation and apoptosis resistant in HCC cells (*P* < 0.05, Fig. 7b-f). Conversely, T0070907 (50 μM), an antagonist of PPAR-γ, rescued the effects of miR-1468 knockdown on biological function of HCC (*P* < 0.05, Fig. 7b-f) in miR-1468-suppressive MHCC-97 L cells. Moreover, alternation of PPAR-γ also abolished the effects of miR-1468 on cell cycle and apoptosis-related proteins (P < 0.05, Fig. 7g). In conclusion, our results indicate that PPAR-γ/AKT signaling plays an essential role in miR-1468-induced HCC growth.

**Fig. 7:** PPAR-γ/AKT signaling is essential for the biological function of miR-1468 in HCC. **a** Hep3B and MHCC-97 L cells that were transfected with corresponding miRNA vectors were subjected to immunoblotting for phosphorylated AKT and AKT. PPAR-γ agonist rosiglitazone treatment inhibited the promotive effects on cell proliferation (**b**, **c**), colony formation (**d**), cell cycle progression (**e**) and apoptosis (**f**) of miR-1468 overexpressing Hep3B cells. PPAR-γ antagonist, T0070907, reversed the suppressive effects of miR-1468 knockdown in MHCC-97 L cells. **g** Western blot analysis indicated that modulating PPAR-γ activation reversed the effects of miR-1468 alteration on cell cycle and apoptosis associated factors of HCC cells. *P < 0.05

### AKT phosphorylation is critical for the biological effects of miR-1468 in HCC

Previous studies report that PPAR-γ exerts its function by inhibiting activation of AKT signaling pathway [30, 31]. To confirm that AKT phosphorylation contributes to the biological function of miR-1468 in HCC cells, we used AKT inhibitor MK2206 or AKT activator IGF-1 (insulin-like growth factor 1) to alter AKT activation. Inactivation of AKT phosphorylation by MK2206 in miR-1468-overexpressing Hep3B cells significantly decreased cell proliferation, cell cycle progression, colony formation (*P* < 0.05, Fig. 8a-d) and induced apoptosis (*P* < 0.05, Fig. 8e). In addition, AKT phosphorylation activator, IGF-1, increased cell proliferation, cell cycle progression, colony formation and inhibited apoptosis (*P* < 0.05, respectively, Fig. 8a-e) in MHCC-97 L-anti-miR-1468 cells. Accordingly, the expression of cell cycle and apoptosis-related proteins were also significantly changed after p-AKT alteration (*P* < 0.05, Fig. 8f). Taken together, our results demonstrate that AKT phosphorylation exerts an important role in miR-1468-mediated HCC grwoth.

**Fig. 8:** AKT phosphorylation is essential for the biological function of miR-1468 in HCC. AKT inhibitor MK2206, or AKT phosphorylation activator IGF-1, abolished the cell proliferation (**a**, **b**), colony formation (**c**), cell cycle progression (**d**) and apoptosis (**e**) of HCC cells which were transduced of miR-1468 vectors. **f** Western blot analysis indicated that modulating AKT phosphorylation reversed the effects of miR-1468 alteration on cell cycle and apoptosis associated factors of HCC cells. *P < 0.05

## Discussion

Increasing evidence confirm that dysregulation of miRNAs plays a critical role in cancer initiation, development and progression, including HCC [32]. Recently, miRNAs have been recognized as diagnostic, therapeutic and prognostic markers [33, 34]. In present study, we confirmed that miR-1468 was up-regulated in HCC tissues and cell lines, which was consistent with TCGA data. Moreover, increased miR-1468 level was obviously correlated with malignant clinicopathological features, including large tumor size, high histological grade and advanced tumor stage. Moreover, miR-1468 was an independent prognostic factor in predicting survival of HCC patients. These data suggest that miR-1468 is involved in HCC progression and represents as a promising biomarker for HCC therapy.

Previous study has confirmed that blood-based circulating miR-1468 is evaluated as a diagnostic marker panel for early diagnosis of pancreatic cancer [15]. In this study, we demonstrated that miR-1468 promoted cell proliferation, cell cycle progression, colony formation and inhibited apoptosis by gain- and loss-of function experiment in vitro and in vivo. Moreover, we provided the first evidence that the target genes of miR-1468 were CITED2 and UPF1. First, miR-1468 negatively modulated CITED2 and UPF1 expression in HCC cells. Second, miR-1468 affected the luciferase activity of wt 3’UTR but not mt 3’UTR of CITED2 and UPF1. Third, miR-1468 was inversely correlated with the expression of CITED2 and UPF1 in HCC tissues. Furthermore, CITED2 and UPF1 were down-regulated in HCC tissues, and modulating their expression could reverse the biological function of miR-1468 in HCC cells. CITED2 is a transcriptional co-regulator that directly interacts with host of transcription factors and co-activators, and influences the activation of gene transcription [35, 36]. CITED2 is a potent prognostic predictor and associated with proliferation, migration and chemoresistance in breast cancer [37]. Moreover, CITED2 serves as a coactivator of hepatocyte nuclear factor 4α (HNF4α) in liver development [38]. CITED2 is a novel direct effector of PPAR-γ in suppressing HCC cell growth [29]. UPF1 is essential for accomplishing DNA replication during S phase of cell cycle [39]. The human RNA surveillance factor UPF1 inhibits hepatic cancer progression and EMT progress by targeting MRP2/ABC2 [40]. Moreover, UPF1 regulates HCC tumorigenesis by up-regulation of SMAD family member 7 (Smad7) and affecting transforming growth factor β (TGF-β) pathway [41]. In this research, we also confirmed that CITED2 and UPF1 were down-regulated in HCC tissues compared to adjacent non-tumor tissues. These data provide more evidence for establishing therapeutic strategies in miRNA-modulating networks.

Previous study reveals that the target genes of miR-1468 are enriched in PPAR signaling pathway [16]. CITED2 signals through PPAR-γ to regulate death of cortical neurons after DNA damage [30]. Moreover, CITED2 is a novel effector of PPAR-γ in inhibiting HCC cell growth [29]. In HCC, PPAR-γ inhibits cell invasion by up-regulating plasminogen activator inhibitor-1. The PPAR-γ agonist has been shown to inhibit HCC development. In this study, alteration of PPAR-γ activation could abolish the effects of miR-1468 on HCC growth. Moreover, PPAR-γ exerted its biological function through AKT signaling. Here, AKT phosphorylation was critical for the biological effects of miR-1468 in HCC. Taken together, we confirm that miR-1468 promotes HCC cell growth by modulation of PPAR-γ/AKT signaling (Additional file 3: Figure S3).

In summary, we demonstrate that miR-1468 overexpression acts as an independent biomarker for indicating poor prognosis of HCC patients. Furthermore, we confirm that miR-1468 promotes cell proliferation, colony formation, cell cycle progression and inhibits apoptosis by directly targeting CITED2 and UPF1 mediated PPAR-γ/AKT pathway. Our data reveal a novel role for miR-1468 in HCC development and progression, and suggest miR-1468 as a potential target for HCC diagnosis and treatment.

## Conclusions

To conclude, our data offer the promising evidence that miR-1468 overexpression acts as an independent risk factor for indicating poor prognosis of HCC patients. miR-1468 facilitates HCC cell proliferation and cell cycle progression, and induces apoptosis in vitro and in vivo. More significantly, CITED2 and UPF1-mediated PPAR-γ/AKT pathway may be directly implicated in the oncogenic function of miR-1468 in HCC. Our study considers miR-1468 as a potential diagnostic marker and therapeutic target for HCC.

## Additional files

Additional file 1: **Figure S1.** Modulation of CITED2 or UPF1 mimics miR-1468-induced cellular processes in HCC. (A) Hep3B-miR-control cells that were transfected with empty vector (EV) or CITED2, UPF1 overexpression plasmid were subjected to western blot for CITED2 and UPF1. MHCC-97 L-anti-miR-NC cells that were transfected with scrambled siRNA or CITED2, UPF1 siRNA were subjected to western blot for CITED2, UPF1. CITED2 or UPF1 restoration mimics the effects of miR-1468 knockdown on cell proliferation (B, C), colony formation (D), cell cycle progression (E) and apoptosis (F) of Hep3B cells. CITED2 or UPF1 knockdown mimics effects of miR-1468 overexpression in MHCC-97 L cells (B-F). (G) Alteration of CITED2 or UPF1 mimics the effects of miR-1468 on cell cycle and apoptosis associated factors. *P < 0.05. (TIFF 704 kb)

Additional file 2: **Figure S2.** CITED2 or UPF1 overexpression promoted PPAR-γ expression and inhibited AKT phosphorylation in HCC cells. (TIFF 1034 kb)

Additional file 3: **Figure S3.** Overview of miR-1468-induced tumor progression and activates PPAR-γ-mediated AKT signaling in human hepatocellular carcinoma. (TIFF 77 kb)

## Abbreviations

CCK-8: Cell Counting Kit-8
CITED2: Cbp/p300 interacting transactivator with Glu/Asp rich carboxy-terminal domain 2
HCC: Hepatocellular carcinoma
HNF4α: Hepatocyte nuclear factor 4α
IF: Immunofluorescence
IHC: Immunohistochemistry
miRNAs: microRNAs
PI3K: Phosphatidylinositol 3-kinase
PPAR-γ: Peroxisome proliferator-activated receptor-γ
pRCC: papillary renal cell carcinoma
qRT-PCR: real-time quantitative reverse transcription polymerase chain reaction
RRM1: Ribonucleotide reductase large subunit M1
TCGA: The Cancer Genome Atlas
TGF-β: Transforming growth factor β
UPF1: Up-frameshift protein 1
